# The Value of CT Three-Dimensional Reconstruction in Nursing and Diagnosis of Senile Hip Fracture

**DOI:** 10.1155/2021/7865155

**Published:** 2021-08-19

**Authors:** Yuanyuan Shi, Si Chen, Xue Chen, Pan Xue

**Affiliations:** ^1^Department of Nursing, The Second Hospital of Jilin University, Changchun 130041, China; ^2^Geriatric Medicine, The Second Hospital of Jilin University, Changchun 130041, China; ^3^Department of Orthopedics, The Second Hospital of Jilin University, Changchun 130041, China

## Abstract

**Aim:**

To study the diagnostic effect of hip fracture in the elderly. In this paper, a total of 100 elderly patients with hip fracture from January 2020 to May 2021 were selected for X-ray and CT examination after admission. The operation was taken as the final criteria for determining hip fracture type, and the diagnosis of hip fracture by CT three-dimensional reconstruction was analyzed and studied. The results showed that the diagnostic rate of CT 3D reconstruction for various types of hip fracture in the elderly was higher than that of CT plain scan and X-ray (*P* < 0.05). For the diagnosis of intra-articular small bone fragments, the rate of missed diagnosis was 2% (2/100) with CT 3D reconstruction, 10% (10/100) with conventional CT scan, and 20% (20/100) with X-ray. The rate of misdiagnosis was 5.0% (5/100) with CT 3D reconstruction. Routine CT scan was 15% (15/100), X-ray was 30% (30/100), and CT 3D reconstruction was significantly lower than other examinations (*P* < 0.05).

**Conclusion:**

CT 3D reconstruction has high accuracy in the diagnosis of various types of hip fractures in the elderly.

## 1. Introduction

Artificial hip arthroplasty has developed for nearly half a century since its development. At present, this technology has become a method for the treatment of hip diseases such as femoral neck fracture, hip osteoarthritis, femoral head necrosis, rheumatoid hip arthritis, ankylosing spondylitis complicated with hip ankylosis, congenital acetabular dysplasia, and hip tumor, It is an effective means to relieve hip pain, restore joint activity, and improve joint stability. It is an effective means to restore joint motion and improve joint stability. Artificial hip replacement includes total hip arthroplasty (THA), total hip replacement (THR), and artificial femoral-head replacement (AFR) [1]. According to statistics, more than 1 million cases of artificial hip arthroplasty have been carried out globally every year, and the number of THA is increasing year by year. By 2015, 0.83% of the total population of the United States has received artificial hip arthroplasty, and the number of artificial hip arthroplasty in China is as high as 200,000 cases every year. At present, the length of hospital stay of patients with hip arthroplasty in China is 13.07 ± 3.49 days, which is generally longer than that of patients in Western countries or regions (5.3 ± 1.6 days). On the one hand, it may be due to the delayed start of functional exercise and getting out of bed. Hip replacement patients, on the other hand, have early postoperative complications such as lower extremity deep vein thrombosis (DVT), infection, postoperative nausea and vomiting (PONV), and prosthesis peripheral fracture. Prolongation of hospitalization time brings an increase in hospitalization costs, increasing the economic burden of medical treatment [2].

Musculoskeletal diseases, including osteoarthritis of the hip and knee, are the second leading cause of disability in almost every country and region in the world, according to a 2010 study on the global burden of disease in the Lancet. The incidence of hip and knee osteoarthritis is increasing year by year worldwide, especially in the elderly population [3]. March et al. have shown that hip diseases, mainly osteoarthritis of the hip, affect nearly 15% of the global population and are a major cause of pain and disability in the elderly. Although there are many treatments available for hip osteoarthritis, joint replacement remains the primary treatment of choice. With the acceleration of population aging process and the development of transportation and construction industry, the incidence of femoral neck fracture increases year by year [4]. Based on data on the incidence of hip fractures, changes in the age composition of the population, and long-term changes in the risk of hip fractures, there are estimates that by 2025, the number of hip fractures will reach 2.6 million (37% in Asia), and by 2050, it will reach 4.5 million (45% in Asia). After China enters the aging society, the incidence of senile fracture increases by 30% every 10 years, and the number of hip fracture also increases at a rate of four times. Hip fractures account for 50% of all fractures caused by osteoporosis in the elderly. Femoral neck fracture is the most common and serious hip fracture. Through retrospective study and comparative analysis, Lee et al. investigated the pelvis of 136 normal adults in order to provide anatomic and morphological data of the coccyx with three-dimensional images for the diagnosis of idiopathic coccygeal pain. Computed tomography used software to reconstruct a three-dimensional model of the pelvis from X-ray images of all the specimens. Unilateral or bilateral fusion of the sacral and coccygeal angles is not uncommon. As far as the transverse processes of sacrum and coccyx are concerned, the separation type is more than the fusion type. The incidence and angle of coccyx deviation vary greatly from individual to individual. A three-dimensional model of the gross anatomy of the coccyx will help to understand the mechanisms underlying the development of idiopathic coccygeal pain [5]. Morgagni hernias can be diagnosed in different ways, but they are not always 100% accurate. A three-dimensional reconstruction of the model may help to better understand important anatomical structures. Zhang et al. performed laparoscopic repair based on a three-dimensional reconstruction model. This case demonstrates that the three-dimensional reconstruction model is a useful tool for the diagnosis and preoperative evaluation of MH patients, especially when the diagnosis is confused in clinical practice [6]. In recent years, with the aging of China's social population, the improvement of people's requirements for the quality of life, the continuous improvement of the medical insurance system, and the rapid development of medicine, the demand for hip replacement in China has increased significantly. It has been more than ten years since ERAS was introduced into China. Through continuous exploration and practice by scholars, remarkable achievements have been made [7]. 2015 was the year of rapid development of ERAS, and the first ERAS collaboration group was established in China. The first ERAS national conference was held in Nanjing in July; the consensus of Chinese experts on the application of accelerated rehabilitation surgery in colorectal surgery (2015 Edition) was released, which includes 19 perioperative measures, mainly including shorten the preoperative ban drink, multimodal analgesia, early postoperative fasting time bed, early to eat drink, restrictive transfusion and minimally invasive surgical operation, the consensus for our country the first ERAS expert consensus. Since then, Chinese scholars have successively published the consensus of ERAS experts in many surgical fields. Including the GanDanYi surgery accelerate rehabilitation expert consensus (2015 edition), the biliary tract surgery accelerate rehabilitation surgery expert consensus (2016 edition), the stomach gastric resection surgery accelerate rehabilitation surgery expert consensus (2016 edition), the laparoscopic hepatectomy accelerate rehabilitation surgery expert consensus (2017 edition),” “China accelerated rehabilitation surgery perioperative tube Consensus of Science Experts (2016 Edition), etc. A systematic evaluation of the application status of ERAS in China shows that ERAS can effectively shorten the length of stay, reduce hospitalization costs, reduce postoperative complications, improve patient satisfaction, improve prognosis and improve the quality of medical care in the surgical fields of gastrointestinal surgery, hepatobiliary surgery, cardiothoracic surgery, urology and obstetrics and gynecology. However, there are still few reports on the application of this advanced surgical concept and technology in the field of orthopedics, especially in hip arthroplasty, and there is still a large research space at present [8].

The innovation point of this paper is that CT 3D reconstruction can not only clearly show the situation of joint fracture, but also select the best Angle of observation of fracture through rotation Angle. In addition, 3D reconstruction can effectively observe the situation of bone fragments, which is conducive to the judgment of hip fracture type and the formulation of surgical plan. The results of this study fully prove that CT examination has a high sensitivity to fracture.CT 3D reconstruction has a high accuracy in the diagnosis of various types of hip fractures in the elderly.

## 2. Materials and Methods

### 2.1. General Information

There were 100 cases in this study, including 53 males and 47 females. The average age was (75.06 ± 2.33) years from 61 to 82 years old. The time from hip injury to admission to hospital ranged from 5 to 52 hours (19.49 ± 6.32) hours on average. Causes of injury: traffic accident injury 45 cases, falling injury 30 cases, fall and fall injury 25 cases. Inclusion criteria: ① All the elderly patients were over 60 years old; ② The symptoms of hip fracture were obvious on admission; ③ All patients had a history of hip trauma before admission; ④ All patients were finally treated by surgery, and the type of hip joint injury was determined by surgery. ⑤ All the patients and their family members agreed to participate in this study, and signed the surgical consent and informed consent. Exclusion criteria: ① Involuntary participation in the study; ② Old or pathological hip fracture; ③ Mental disorders can not take the initiative to participate in surgical treatment.

### 2.2. Examination and Treatment Methods

① X-ray examination: the machine model is Siemens YSIO, and the hip joint and pelvis are scanned in the positive position.
② CT examination: CT models were Siemens SOMATOMdefinionAS and GebrightSpeed, scanning from both iliac wings to ischial nodular, voltage: 120 kV, current: 90 mA, matrix: 512 × 512, layer thickness: 2.5 mm, field: 400 × 400 mm.
③ CT three dimensional reconstruction: 1∼1.25 mm, with a thick layer of layer spacing of 1 mm, relevant data import post-processing software, multiplanar reconstruction (MPR), bone reconstruction algorithm was used to rebuild, according to the direction of horizontal, vertical axis coordinates of human body adjust, select effective fracture plane imaging, further analyze the fracture type, form, and so on and so forth. Surgical treatment: ① Joint replacement for femoral neck fracture; ② Femoral trochanteric fracture should be treated with proximal femoral anti-rotation intramedullary nail; ③ Acetabular fractures were treated with open reduction plate fixation.

### 2.3. To Observe

Using surgery as the final criteria to determine the type of hip fracture, we compared the diagnosis of various types of hip fracture with X-ray, conventional CT scan and CT three-dimensional reconstruction. Two attending radiologists read the radiographs respectively. When the results were inconsistent, the same conclusion could be reached after joint discussion.

### 2.4. Statistical Method

SPSS18.0 data statistical software was used to establish a database and statistical analysis was conducted. Measurement data was expressed as (*x* ± *s*), enumulation data as rate (%), *χ*2 test was used for comparison, *P* < 0.05, which was statistically significant.

The materials and methods section should contain sufficient detail so that all procedures can be repeated. It may be divided into headed subsections if several methods are described.

## 3. Results and Discussion

### 3.1. The Diagnosis of Various Types of Senile Hip Fractures by Different Examination Methods

The diagnosis of various types of senile hip fracture by different examination methods: in 80 cases of senile hip fracture patients, conventional CT scan and CT three-dimensional reconstruction were completely detected (100.0%), and the detection rate of X-ray examination was 81.25% (81.25/100), the difference was statistically significant(*χ*2 = 5.2396, *P* > 0.05); In this study, 117 hip fractures were found, including 58 femoral neck fractures, 29 intertrochanteric fractures, and 30 acetabulum fractures. In the acetabular fractures, 5 anterior wall, 8 posterior wall, 6 anterior column, 7 posterior column and 4 acetabular floor were involved. The detection rate of CT three-dimensional reconstruction for femoral neck fracture, intertrochanteric fracture and acetabular fracture was higher than that of conventional CT scan and X ray (*P* < 0.05). See Table 1.

### 3.2. Diagnosis of Intra-Articular Small Bone Fragments by Different Examination Methods

Different examination methods for the diagnosis of intraarticular small bone fragments: For the diagnosis of intraarticular small bone fragments, the rate of missed diagnosis was 2% (2/100) with CT 3D reconstruction, 10% (10/100) with conventional CT scan and 20% (20/100) with X-ray. The rate of misdiagnosis was 5.0% (5/100) with CT 3D reconstruction. Routine CT scan was 15% (15/100), X-ray was 30% (30/100), CT 3D reconstruction was significantly lower than other examinations (*P* < 0.05). See Table 2.

## 4. Conclusions

The acetabulum, femoral head and other tissues together constitute the hip joint, which can cause hip injury when it is subjected to the external force of several times the weight of human body. Since osteoporosis is common in older people, mild violence can lead to hip fractures. Because of the decline in the metabolism of the elderly patients themselves, the recovery time is prolonged after the trauma, and in severe cases, other serious concurrent diseases will be caused. For the elderly patients with hip fracture, timely diagnosis and treatment is very important. CT examination has the characteristics of short time and quick scan, and can collect volumetric data at the same time, the thickness of the layer is extremely thin. CT post - processing technology can obtain three - dimensional images. In addition, the examination results of various types of hip fractures in this study showed that CT three-dimensional reconstruction had the highest diagnostic rate for femoral neck, intertrochanteric and acetabular fractures. Because hip fracture is often accompanied by bone fragments displaced, some of the bone fragments are easy to embed in the joint, and it is not easy to be observed in the examination process. In severe cases, it can lead to necrosis of the femoral head or arthritis, which can affect the prognosis of elderly patients to a certain extent. The results of this study effectively proved the advantage of 3D reconstruction in the diagnosis of small intraarticular bone fragments. Multi-plane reconstruction can clearly display the femoral head and acetabulum, and observe the joint fracture from multiple angles. Higher tissue resolution can improve the recognition of small fragments of bone, and further improve the diagnosis rate of hip fracture. In conclusion, CT 3D reconstruction has a high accuracy in the diagnosis of various types of hip fractures in the elderly.

## Figures and Tables

**Table 1:** The diagnosis of various types of senile hip fractures by different examination methods.

The fracture types	CT 3D reconstruction	Routine CT	X-ray
Femoral neck fracture	100.0% (58/58)	94.83% (55/58)	86.21% (50/58)
Intertrochanteric fracture of femur	100.0% (29/29)	93.10% (27/29)	75.86% (22/29)
Acetabulum fracture	96.67% (29/30)	86.67% (26/30)	56.67% (17/30)

*Note*. ① Femoral neck fracture: Comparison of 3D reconstruction and conventional CT, *χ*2 = 4.1039, *P* < 0.05; Three-dimensional reconstruction compared to X-ray, *χ*2 = 7.6631, *P* < 0.05; Conventional CT versus X-ray, *χ*2 = 6.0583, *P* < 0.05; ② Intertrochanteric fracture of femur: comparison of three-dimensional reconstruction and conventional CT, *χ*2 = 5.2043, *P* < 0.05; Three-dimensional reconstruction compared to X-ray, *χ*2 = 11.0926, *P* < 0.05; Conventional CT versus X-ray, *χ*2 = 9.2235, *P* < 0.05; ③ Acetabular fractures: Comparison of 3D reconstruction and conventional CT, *χ*2 = 8.4921, *P* < 0.05; Three-dimensional reconstruction compared to X-ray, *χ*2 = 16.3928, *P* < 0.05; Conventional CT versus X-ray, *χ*2 = 12.1149, *P* < 0.05.

**Table 2:** Diagnosis of intraarticular small bone fragments by different examination methods.

The fracture types	The missed diagnosis (%)	The misdiagnosis rate (%)
CT 3D reconstruction	2.5	5.0
Routine CT	8.75	12.50
X-ray	18.75	27.50

*Note*. In terms of missed diagnosis rate, the comparison between CT 3D reconstruction and conventional CT, *χ*2 = 3.3649, *P* < 0.05; Comparison of CT 3D reconstruction and X-ray, *χ*2 = 8.0237, *P* < 0.05; Routine CT scans compared to x-rays, *χ*2 = 5.1282, *P* < 0.05; In terms of misdiagnosis rate, the comparison between CT 3D reconstruction and conventional CT, *χ*2 = 3.4035, *P* < 0.05; Comparison of CT 3D reconstruction and X-ray, *χ*2 = 11.2391, *P* < 0.05; Routine CT scans compared to x-rays, *χ*2 = 8.0907, *P* < 0.05.

## Data Availability

The data used to support the findings of this study are available from the corresponding author upon request.
